RETRACTED

# CRNDE/ETS1/GPR17 Facilitates the Proliferation, Migration, and Invasion of Glioma

**DOI:** 10.1155/2021/7566365

**Published:** 2021-10-26

**Authors:** Yan Hu, Haitao Luo, Xingen Zhu, Hua Guo

**Affiliations:** ^1^Department of Neurosurgery, The Second Affiliated Hospital of Nanchang University, Nanchang, Jiangxi Province 330006, China; ^2^East China Institute of Digital Medical Engineering, Shangrao, Jiangxi Province 334000, China; ^3^Institute of Neuroscience, Nanchang University, Nanchang, Jiangxi Province 330006, China

## Abstract

**Background:**

Numerous lncRNAs were found as regulatory factors for occurrence and progression of various tumors, but there is still less research on the role of lncRNAs in malignant progression of glioma.

**Methods:**

Bioinformatics analysis analyzed differential genes (DEGs) in the TCGA database. MTT, flow cytometry, and Transwell assays were performed to test the proliferation, apoptosis, migration, and invasion of cells. qRT-PCR and western blot were conducted to detect RNA and protein expressions of each gene, respectively. CHIP assay verified the binding relationship between genes. FISH assayed subcellar location of CRNDE, and xenograft in nude mice was performed for *in vivo* verification.

**Results:**

CRNDE was upregulated in glioma cells, and overexpression of CRNDE facilitated malignant progression of glioma cells. CRNDE regulated occurrence and development of glioma through the CRNDE-ETS1-GPR17 axis. ETS1 was proved to target promoter region of GPR17. Overexpression of CRNDE promoted the binding between ETS1 and the promoter region of GPR17, thus, promoting the transcription of GPR17, while silencing of GPR17 inhibited promotion of CRNDE on proliferation, migration, and invasion of glioma cells.

**Conclusions:**

These results demonstrated that CRNDE regulated GPR17 expression by binding ETS1, a transcription factor, thereby affecting glioma development. The results also indicated that CRNDE could serve as a possible therapeutic target and prognostic biomarker for glioma.

## 1. Introduction

Glioma is an aggressive primary brain tumor, which is featured as invasive growth and early metastasis [1]. Glioblastoma multiforme (GBM) is the predominant subtype of all types of glioma with a survival rate generally less than 5 years [2]. The high recurrence rate and low treatment efficiency of glioma lead to poor prognosis. Although surgical resection, radiotherapy, chemotherapy, and targeted therapy have developed in recent decades, the treatment of glioma, especially GBM, is still not satisfactory [3]. Development of glioma is complex, which is accomplished by multigene interaction and multimolecule regulation [4]. It is vital to study molecular mechanism of glioma for effective avenues and prognosis methods of glioma.

lncRNAs have become a research hotspot due to its aberrant expression in various tissues, particularly in tumor tissues [5–8]. Recent studies display that lncRNAs participate in varying biological processes in the human body, such as transcriptional activation of cells, intracellular transport, heat shock response, and genomic imprinting [9–11]. lncRNAs are associated with various malignant tumors and exist in tumors as oncogenes and prooncogenic factors [12]. There are also some reports on the impacts of lncRNAs on proliferation and metastasis of glioma. Yan et al. have discovered that lncRNA FlvCR1-AS1 modulates E2F2 level by competitive adsorption of miR-4731-5p, further promoting proliferation and metastasis of glioma [13]. A study of Li et al. proves that downregulation of LINC00174 can inhibit resistance to temozolomide in the glioma cells, the molecular mechanism of which is that LINC00174 can sponge miR-138-5p so as to affect the expression of SOX9 and further improves the resistance to temozolomide and proliferation of glioma cells [14]. In addition to serving as ceRNAs to further regulate the biological function of glioma through competitive adsorption of miRNAs, lncRNAs can also directly regulate gene expression in combination with transcription factors to influence the development of glioma. Lv et al. found that lncRNA PVT1 can promote proliferation and migration of glioma cells by downregulating the expression of UPF1 [15]. However, the specific molecular mechanism of lncRNAs on glioma progression, especially the regulation of lncRNAs in combination with transcription factors on glioma progression, needs to be further explored.

RETRACTED

As a lncRNA, CRNDE exerts an essential role in a variety of cancers. Sun et al. reported that CRNDE promotes the chemosensitivity of medulloblastoma cells via modulating miR-29c-3p level [16]. Bai et al. demonstrated that CRNDE as an oncogene in cervical cancer could promote the development of cervical cancer via increasing CCNB1 level by competitively adsorbing miR-183 [17]. These reports confirm the importance of CRNDE in cancer development. CRNDE functions in development of glioma. Li et al. put forward that CRNDE as a ceRNA facilitates progression of GBM via modulating miR-136-5P/Bcl-2/Wnt2 signal axis [18]. Kiang et al. found that CRNDE functions in promoting glioma progression, while the promoting effect is regulated by EGFR signal [19]. These studies on glioma have proved the effect of CRNDE on glioma, but the specific molecular mechanism of CRNDE regulating glioma still needs further research, especially whether it can combine relevant transcription factors to regulate downstream genes, thus, affecting the development of glioma.

RETRACTED

The study committed to studying relationship between CRNDE and the progression of glioma and to probing into the impact of CRNDE on biological behavior of glioma cells and the possible molecular mechanism of CRNDE binding to transcription factors to regulate downstream genes, so as to shed new light on targeted therapy for glioma. In this study, we used bioinformatics methods to demonstrate that CRNDE was differentially expressed between normal and tumor tissues and to screen possible downstream genes regulated by CRNDE. ETS1/GPR17 was selected for further study. Finally, the lncRNA-TF-mRNA regulatory axis of CRNDE was verified by bioinformatics and related experiments. Our study may provide new insights into pathogenesis of glioma and uncovering of novel therapeutic targets.

## 2. Materials and Methods

### 2.1. Bioinformatics Analysis

Relevant lncRNAs of glioma were from LINCDISEASE (http://www.rnanut.net/lncrnadisease/index. html), and lncRNAs with detection methods of Experimental and Experimental/Predicted were retained. A glioma expression chip GSE50161 (normal: 13; tumor: 34) was acquired from GEO (https://www.ncbi.nlm.nih.gov/GEO/). Differential analysis was completed by using R package “limma” with normal samples as controls. ∣logFC | >2 and *P* value < 0.05 were used as the screening criteria for the differential lncRNAs (DElncRNAs) and mRNAs (DEmRNAs). CRNDE, ETS1, and GPR17 levels in TCGA-LGG were retrieved through GEPIA (http://gepia2.cancer-pku.cn/#index). Downstream transcription factors and triplet for regulating genes of CRNDE in low-grade glioma (LGG) were predicted by using lncMAP (http://bio-bigdata.hrbmu.edu.cn/ lncMAP/survival. JSP). The jasper database was employed to predict binding sites of ETS1 and promoter regions of downstream genes.

### 2.2. Cells and Cell Culture

Cell line information was listed in Table S1. Normal HEB cells and glioma cells T98G, A172, SNB19, and U251 were prepared in a complete Dulbecco's modification of Eagle's medium (DMEM; Sigma, USA) containing 10% fetal bovine serum (FBS; NY, USA) and with addition of 100 U/mL penicillin/streptomycin (Corning, NY, USA) in an incubator under standard conditions.

### 2.3. Cell Transfection

Full-length sequence of CRNDE was cloned, and the vectors of CRNDE overexpression (oe-CRnDE) and blank pcDNA3.1 (oe-NC) were constructed from GENECHEM, Shanghai. Sh-ETS1 and its control (sh-NC), sh-GPR17 and its control (sh-ctrl) sequences were accessed from RiboBio (China). T98G and U251 cells were transfected for 48 h for subsequent analysis. pLent-CRNDE and pLent-NC vectors were purchased from Vigene Biosciences (USA) and used for lentivirus transduction of overexpressed CRNDE. Lentivirus vectors were transfected into T98G cells and treated with 1 mg/mL puromycin to obtain stable cell lines. Cell transfection was completed with Lipofectamine 3000 (L3000015, Invitrogen, USA).

RETRACTED

### 2.4. qRT-PCR

Total RNA isolation from tissue and cells of each group was completed using Trizol (Invitrogen) following manufacturer's guidelines. The PrimeScript™ RT reagent Kit (TakaRa, Shiga, Japan) was recommended for reverse of cDNA. qRT-PCR was done on an ABI 7900HT instrument (Applied Biosystems, USA). Quantitative PCR was done on SYBR Premix Ex Taq (TaKaRa, Otsu, Shiga, Japan). CRNDE was normalized with 36B4 as endogenous control. ETS1 and GPR17 were normalized with GAPDH as endogenous control. Primers were listed in Table S2. The differences in relative level of target gene in the control group and experimental group were compared by 2^-*ΔΔ*Ct^ value. The assay was conducted in 3 replicates.

### 2.5. Western Blot

48 h after cells were transfected in various groups, they were rinsed with cold PBS (Thermo Fisher, USA) in triplicate and lysed on ice for 10 min with whole protein lysate. Protein quantification was done with BCA quantitative kit (Thermo Fisher, USA). 10 *μ*L loading buffer was supplemented, and proteins were boiled for 10 min at 95°C. SDS-PAGE was performed at 100 V. After the electrophoresis, proteins were transferred to the NC membrane at 100 mA and 120 min, sealed with 5% BSA/TBST for 60 min, followed by incubation with primary antibodies at 4°C overnight. After incubation, the membrane was washed in a shaking table with 1 × TBST solution (Solarbio, Beijing, China) 5 min × 3 times at room temperature. Goat anti-rabbit IgG labelled with horseradish peroxidase was used for hybridization for 120 min at room temperature. Membrane was washed with TBST for 20 min × 3 times and. Then, luminescence reaction was performed with ECL kit (Solarbio, Beijing, China). Protein imprinting was observed by taking photos. The assay was done in three replicates. Antibody information was exhibited in Table S3.

### 2.6. Chromatin Immunoprecipitation (CHIP) Assay

T98G and U251 cells were used for CHIP assay. EZ-Magna ChIP (Millipore) kit was recommended in ChIP assay. The experiment was briefly described as follows. First, 1% formaldehyde solution was applied to the cells to induce cross-linking. Then the cross-linking was quenched with 140 mM glycine. The acquired nucleic acid protein complex was then lysed to 200-500 bp DNA fragments and immunoprecipitation of the experimental antibody or IgG. After 4°C overnight, the cross-linking of DNA was removed, and target fragment level was assayed via qRT-PCR. The primers used in the assay were in Table S2. The antibody information used in the assay was in Table S3.

RETRACTED

### 2.7. MTT Assay

The proliferation of T98G and U251 cells (5 × 10^3^/100 *μ*L) was measured by MTT assay. Each processing consisted of three duplicates. After 24 h of cell culture, 48, 72, 96, and 120 h, sterile MTT solution (Beyotime) was used to assess cell proliferation. Absorbance at 450 nm wavelength was assayed with a microplate reader (Sunnyvale, CA, USA).

### 2.8. Cell Apoptosis Assay

T98G and U251 cells were cultured in a 6-well plate. After 48 h of culture, cells were digested by trypsin (without EDTA) and then re-suspended in PBS (4°C). After centrifuged at 1000 rpm and 4°C to remove PBS, cells were resuspended by using binding buffer (1×). Annexin V-FITC (Biovision, K101) and propidium iodide (PI) staining suspension were added. The response of cells was conducted in dark for 15 min, and proportion of cell apoptosis was assayed by flow cytometry (BD Biosciences).

### 2.9. Transwell Migration and Invasion Assays

T98G and U251 cells in logarithmic growth phase were starved for 24 h, and on the next day, digested cells were centrifuged and resuspended. The final cell concentration was 2 × 10^4^ cells/mL. Transwell upper chamber was supplemented with 0.2 mL suspension, and lower chamber was filled with 700 *μ*L DMEM plus 10% FBS. Cells were prepared in a culture chamber under routine conditions. 24 h later, cells in the upper insert were swabbed with wet cotton swabs. Then, cells were subjected to fixing with methanol for 30 min and staining with 0.5% crystal violet for 20 min. In the invasion assay, the final cell concentration was 1 × 10^4^ cells/mL, and the Matrigel-coated upper chamber was recommended. DMEM plus 10% FBS was used to fill the lower chamber. The cells were incubated at 37°C for 48 h and then stained with crystal violet for 20 min. The stained cells in these two assays were washed with PBS and dried upside-down. Then, cells were photographed under an inverted microscope. Five fields were randomly chosen for counting cells.

### 2.10. Fluorescence In Situ Hybridization (FISH) and Subcellular Fractionation

For FISH assay, first, the fluorescent probe was synthesized on CRNDE, which was purchased from RiboBio (Guangzhou, China). Afterward, Ribo FISH Kit and Ribo lncRNA FISH Probe Mix Kit were used to perform FISH assay (RiboBio, Guangzhou, China) on brain glioma tissues in accordance with the instructions. After the assay, the fluorescent microscope was used to observe the results (Thermo Fisher, USA) and photographed. The cell nucleus and cytoplasm of T98G and U251 were extracted with PARIS Kit according to the kit specifications (Life Technologies, Carlsbad, USA). After the separation, the expressions of CRNDE and reference genes (U6 and GAPDH) in the cell nucleus and cytoplasm were assayed via qRT-PCR.

RETRACTED

### 2.11. Statistical Analysis

Data were handled by SPSS 22.0 (Chicago, IL, USA). Measurement data were expressed as mean ± standard deviation. The comparison between two groups was *t*-test, and the comparison between multiple groups was one-way ANOVA. The chi-square test was used for CRNDE and clinicopathological parameters. *P* < 0.05 indicated a statistically significant difference, while *P* < 0.01 and *P* < 0.001 indicated an extremely significant difference.

## 3. Results

### 3.1. CRNDE Expression Is Increased in Glioma

In order to search for DELncRNAs associated with glioma, 142 glioma-related lncRNAs were screened from the LINCDISEASE database. 37 DelncRNAs were obtained through limma differential analysis of GSE50161 chip from the GEO database. Five DElncRNAs including MEG3, CRNDE, XIST, AgAP2-AS1, and LINC01116 that were related to glioma were obtained by taking the intersection of DElncRNAs and glioma-related lncRNAs (Figure 1(a)). By analyzing the expression differences of these 5 lncRNAs in normal samples and glioma tumor samples of GSE60161 chip, CRNDE was significantly upregulated in tumor samples (Figure 1(b)), and the difference was the most significant when compared with the normal samples (∣logFC | = 4.342887) (Table S4). CRNDE has been reported to foster occurrence of colorectal cancer, breast cancer, and other cancers [20, 21]. However, no studies on the impact of CRNDE on glioma and molecular mechanism have been reported, so we chose CRNDE as the research object for subsequent studies. Since there was no normal tissue data for GBM in the TCGA database, we compared the clinical expression data of CRNDE in the GEPIA database. The results exhibited that CRNDE was significantly upregulated in LGG tumor samples (Figure 1(c)), which was basically congruous with CRNDE trend in the GEO database.

CRNDE level in HEB cells and glioma cells T98G, A172, SNB19, and U251 was assayed via qRT-PCR. The results were that CRNDE was markedly highly expressed in all 4 glioma cell lines when compared to HEB cells (Figure 1(d)). These results displayed that CRNDE was upregulated in glioma cells. T98G and U251 were the cell lines with the highest and lowest CRNDE expression in the 4 cancer cell lines, respectively, so they were chosen for the following *in vitro* cell experiments.

### 3.2. Overexpression of CRNDE Modulates Proliferation, Apoptosis, Migration, and Invasion of Glioma Cells

From CRNDE level in clinical tissue and cells, it could be concluded that CRNDE level was positively correlated with tumor occurrence. Therefore, it is inferred that forced expression of CRNDE in glioma cells would promote proliferation, migration, and invasion of cancer cells. To verify the possibility, we examined the impacts of the forced CRNDE expression on malignant behaviors of T98G and U251 cells. MTT and cell apoptosis assays denoted that enforced CRNDE expression noticeably promoted viability, growth abilities, and inhibited apoptosis of both cells (Figures 2(a) and 2(b)). In addition, we also confirmed that CRNDE was expressed in both nucleus and cytoplasm of cancer tissues and cells using FISH assay and nuclear/plasma separation experiment, and the expression level in the nucleus was remarkably higher than that in the cytoplasm (Figure 2(c)). Hence, CRNDE may modulate downstream transcription factors. We further examined the effect of CRNDE on the migration and invasion of glioma cells that were significantly enhanced after CRNDE was overexpressed (Figure 3(a)). Western blot was used to assay invasion- and migration-related proteins, and the results also displayed that the expression levels of N-cadherin, Vimentin, MMP9, and MMP2 increased while that of E-cadherin decreased after CRNDE overexpression (Figure 3(b)). Taken together, CRNDE could act as a prooncogenic factor to modulate proliferative, migratory, invasive, and apoptotic properties of glioma cells, as well as EMT process.

RETRACTED

### 3.3. CRNDE Promotes GPR17 Expression by Promoting Binding of ETS1 to GPR17 Promoter Region

After it was determined that CRNDE facilitated malignant progression of glioma cells, the downstream transcription factors and targeted mRNAs of CRNDE that could regulate glioma cells were explored. We used the lncMAP database to predict the regulatory triplet lncRNA-TF-mRNA of CRNDE in brain glioma and obtain 30 downstream regulatory transcription factors. Four candidate transcription factors, ETS1, MYC, NR3C2, and FOXP2, were obtained by intersecting these 30 transcription factors with significantly DemRNAs in GSE50161 (Figure 4(a)). By analyzing the expression differences of these 4 transcription factors from GSE50161 chip in normal samples and glioma tumor samples, it was noted that ETS1 was remarkably upregulated in tumor samples (Figure 4(b)) with the most prominent difference when compared with the normal samples (∣logFC | = 2.558219) (Table S4). Besides, we compared the mRNA expression data of ETS1 in the GEPIA database, and the results displayed that ETS1 was notably upregulated in the tumor samples of LGG (Figure 4(c)). At the same time, GPR17 was obtained by taking intersection of DElncRNAs in GSE50161 and mRNAs in predicted results of lncMAP triplet (Figure 4(d)). GPR17 expression in GSE50161 chip and GEPIA database clinical data revealed that GPR17 was highly expressed in tumor samples (Figures 4(e) and 4(f)).

RETRACTED

After the regulation pathway of CRNDE-ETS1-GPR17 was found by bioinformatics analysis, multiple experiments were conducted to verify their binding relationship. qRT-PCR detection displayed that forced CRNDE expression would promote GPR17 level in cancer cells (Figure 5(a)). In order to study whether ETS1, bound to the promoter region of GPR17 to regulate the transcription of GPR17, we used the Jaspar database to predict binding sites of ETS1 and GPR17 promoter region, and CHIP along with qRT-PCR assays were used to prove that ETS1 could bind to GPR17 promoter region (Figure 5(b)). Then, the cells were divided into oe − NC + sh − NC, oe − CRNDE + sh − NC, and oe − CRNDE + sh − ETS1 groups. Protein and mRNA expressions of GPR17 in each group were detected, respectively. It was found that silencing ETS1 inhibited the promoting effect of overexpressed GPR17 in two glioma cells (Figures 5(c) and 5(d)). These results demonstrated the mutual binding effect of CRNDE-ETS1-GPR17 and suggested that CRNDE may promote the expression of GPR17 by regulating ETS1.

### 3.4. CRNDE Regulates GPR17 to Modulate the Phenotypes of Glioma Tumor Cells

In order to prove that CRNDE modulated the biological function of glioma through modulating the expression of GPR17, we conducted rescue experiments in T98G and U251 cells. Based on the results of the MTT assay, the cell activity was significantly increased after the overexpression of CRNDE, while promoting ability of CRNDE overexpression was significantly inhibited when GPR17 was inhibited (Figure 6(a)). The results of apoptosis were opposite to the proliferation results. The apoptosis rate of the cells in the oe − CRNDE + sh − GPR17 group was significantly higher than that in the oe − CRNDE + sh − Ctrl group (Figure 6(b)). In terms of cell migration and invasion, overexpression of CRNDE and inhibition of GPR17 would inhibit the promoting effect of CRNDE overexpression on cells (Figure 6(c)). Western blot assayed levels of invasion- and migration-related proteins, and the results also showed that oe − CRNDE + sh − GPR17 reversed the ability of overexpressing CRNDE alone to regulate protein expressions. In other words, protein levels of N-cadherin, Vimentin, MMP9, and MMP2 decreased while that of E-cadherin increased in the reverse group (Figure 6(d)). In summary, CRNDE may foster occurrence and development of glioma cells by promoting GPR17 level.

RETRACTED

## 4. Discussion

Glioma is a kind of destructive and invasive brain tumor and main cause of central nervous system tumor-related death in adults, early diagnosis, and treatment of which are still medical problems. In researches of tumors, lncRNAs participate in varying processes of tumor genesis and exert regulatory roles in occurrence and development of tumors. It is also important to know the biological functions of lncRNAs in the regulation of tumor carcinogenesis and tumor inhibition. CRNDE was speculated to modulate proliferation and metastasis of brain glioma cells through bioinformatics prediction. Bioinformatics prediction and qRT-PCR disclosed that CRNDE was upregulated and may modulate malignant behaviors of glioma cells. Here, CRNDE was upregulated in glioma cells. Hence, we studied the effect of CRNDE on the functions of glioma, and the results exhibited that the forced expression of CRNDE markedly promoted proliferation, migration, invasion, and antiapoptosis of glioma cells. These results all confirmed that CRNDE was a prooncogenic factor in glioma and had a notable promoting impact on the functions of cancer cells.

Numerous reports explained the regulatory impact of lncRNAs on the biological functions of glioma, and most studies in glioma focus on the fact that lncRNAs can bind small RNAs as endogenous sponging small RNAs or competitive endogenous RNAs (ceRNAs) and regulate their functions [22, 23]. In addition to being ceRNAs, lncRNAs in combination with transcription factors to regulate downstream genes to affect glioma function have also been concerned. Li et al. reported that lncRNA HOTAIRM1 foster proliferation and metastasis of GBM by upregulating HOXA1 and inhibiting the binding of HOXA1 to the G9a/EZH2/Dnmts complex [24]. Fei et al. have discovered that lncRNA SNHG3 facilitates the malignant progression of glioma through recruiting zeste homolog 2 enhancer onto promotors of KLF4 and p21 [25]. We unraveled that CRNDE modulated GPR17 level by binding to ETS1, so as to promote glioma malignant progression. This result further confirmed that lncRNAs in glioma could affect the development of glioma by binding some transcription factors to further regulate the expression of downstream mRNAs.

As a member of the ETS family, the function of ETS1 in human body has been extensively studied due to its expression in different cell types. In tumors, it functions by acting on stromal cells and tumor cells in tumor tissues. ETS1 fosters growth of tumor cells and stromal cells in tumor tissues during the development of a variety of tumors [26–29]. Although few studies investigated the role of ETS1 in glioma, previous relevant studies have also proved that ETS1 functions on promoting cancer in glioma. Gabler et al. have put forward that ETS1 functions on promoting the growth of cancer cells in both malignant gliomas and LGG [30]. In this study, we found that ETS1 could be bound by CRNDE to promote levels of downstream mRNAs and enhance the malignant phenotype of glioma cells. On the one hand, these results proved the prooncogenic role of ETS1 in glioma. On the other hand, ETS1 was proved to play an important role as a transcription factor in glioma.

RETRACTED

GPR17 is a G-protein-coupled receptor (GPCR) binding to the Gi subunit, which is mainly confined to the oligodendrocyte lineage cells. GPR17 is critical for the time of myelin formation in oligodendrocytes [31]. The role of GPR17 in cancer is rarely reported. In this study, it was found that GPR17 was located in the regulating lncRNA-TF-mRNA axis of CRNDE-ETS1-GPR17 in glioma by bioinformatics. Further experiments showed that GPR17 could promote the malignant progression of glioma cells, and its modulatory impact was controlled by CRNDE-ETS1. These results displayed for the first time that GPR17 played a prooncogenic role in glioma and the molecular mechanisms by which it was regulated in glioma was also proved.

This study unraveled that CRNDE promoted the development of glioma cells. CRNDE upregulated GPR17 expression in combination with ETS1 to foster proliferation, migration, invasion, and hinder apoptosis of glioma cells. This study generates a deeper understanding of the role of CRNDE in glioma and lays a foundation for seeking new targeted therapies for glioma. We will collect clinical samples and establish mouse models *in vivo* to investigate the relationship between the modulatory axis and clinicopathology of glioma patients or the relationship with tumor metastasis *in vivo*.

## Figures and Tables

**Figure 1:** CRNDE expression is increased in glioma. (a) The Venn diagram of intersection between the DElncRNAs in GSE50161 and glioma-related lncRNAs in LINCDESEASE database. (b) The differential expressions of the five candidate lncRNAs in GSE50161 chip, the *x*-coordinate represents the name of lncRNA, and the *y*-coordinate represents the expression value. Blue box plot represents the normal samples, and the red box plot represents the tumor samples. (c) CRNDE level in LGG in TCGA database, the red box plot indicates tumor samples, and the gray box plot indicates normal samples. (d) CRNDE level in HEB cells and glioma cells T98G, A172, SNB19, and U251 were assayed via qRT-PCR. ^∗^*P* < 0.05, ^∗∗^*P* < 0.01, ^∗∗∗^*P* < 0.001.

**Figure 2:** Overexpression of CRNDE promotes proliferation of glioma cells and the localization of CRNDE in tissues and cells. (a) and (b) MTT and flow cytometry assays assayed the growth activity and apoptosis of T98G and U251 cells after CRNDE overexpression. (c) FISH was used to locate the CRNDE in glioma tissues. Levels of GAPDH (cytoplasmic marker), U6 (nuclear marker), and U251 were measured by qRT-PCR after the nuclear and cytoplasmic separation of T98G and U251 cells. ^∗^*P* < 0.05.

RETRACTED

**Figure 3:** Overexpression of CRNDE fosters migration, invasion, and expression of marker proteins in glioma cells. (a) Transwell assay assessed migratory and invasive abilities of T98G and U251 cells after CRNDE overexpression (100×). (b) Western blot assayed levels of migration- and invasion-related proteins after CRNDE overexpression. ^∗^*P* < 0.05.

**Figure 4:** CRNDE-regulated transcription factors and downstream targeted gene expression. (a) Venn diagram of intersection of CRNDE downstream transcription factors predicted by lncMAP database and DElncRNAs in GSE50161 chip. (b) Differential expression of the four candidate transcription factors in GSE50161 chip, the *x*-coordinate represents the transcription factor name, and the *y*-coordinate represents the expression value. The blue box plot represents the normal samples, and the red box plot represents the tumor samples. (c) ETS1 level in LGG in TCGA database, the red box plot indicates tumor samples, and the gray box plot indicates normal samples. (d) The Venn diagram of the intersection of mRNA in predicted CRNDE-ETS1-mRNA triplet by lncMAP database and DElncRNAs in GSE50161 chip. (e) Differential expression of GPR17 in GSE50161, blue box represents normal samples, and red box represents tumor samples. (f) GPR17 level in LGG in TCGA database, the red box plot indicates tumor samples, and the gray box plot indicates normal samples. ^∗^*P* < 0.05, ^∗∗^*P* < 0.01, ^∗∗∗^*P* < 0.001.

**Figure 5:** CRNDE promotes GPR17 expression by regulating the combination of ETS1 and GRP17. (a) Effect of overexpressed CRNDE on GPR17 level in T98G and U251 cell lines. (b) Binding relationship between ETS1 and GPR17 promoter region in T98G and U251 cell lines was detected by CHIP and qRT-PCR. (c) and (d) Western blot and qRT-PCR assayed protein and mRNA levels of GPR17 in cell lines of each group. ^∗^^#^*P* < 0.05, ^∗^ in Figure 5 represents in comparison with oe − NC + sh − NC, and ^#^ represents in comparison with oe − CRNDE + sh − NC.

**Figure 6:** CRNDE regulates GPR17 to facilitate the malignant progression of glioma tumor cells. (a) and (b) MTT and flow cytometry assays assayed the growth activity and apoptosis of T98G and U251 cells in each treatment group. (c) Transwell assay assessed the migratory and invasive abilities of T98G and U251 cells in each treatment group (100×). (d) Western blot assayed levels of migration- and invasion-related proteins in U251 cells. ^∗^^#^*P* < 0.05, ^∗^ represents in comparison with oe − NC + sh − Ctrl, ^#^ represents in comparison with oe − CRNDE + sh − Ctrl.

RETRACTED

## Data Availability

Please contact corresponding author with reasonable request for the original experimental data and materials.

## Supplementary Materials

Supplementary Materials Table S1: cell lines used in the experiments. Table S2: primer sequences used in the experiments. Table S3: antibody information used in the experiments. Table S4: differential expressions of screened DElncRNAS and transcription factors.
